# Lobeglitazone Attenuates Airway Inflammation and Mucus Hypersecretion in a Murine Model of Ovalbumin-Induced Asthma

**DOI:** 10.3389/fphar.2018.00906

**Published:** 2018-08-08

**Authors:** Na-Rae Shin, Sung-Hyeuk Park, Je-Won Ko, Young-Kwon Cho, In-Chul Lee, Jong-Choon Kim, In-Sik Shin, Joong-Sun Kim

**Affiliations:** ^1^College of Veterinary Medicine BK21 Plus Project Team, Chonnam National University, Gwangju, South Korea; ^2^College of Health Sciences, Cheongju University, Cheongju, South Korea; ^3^Natural Product Research Center, Korea Research Institute of Bioscience and Biotechnology, Jeongeup, South Korea; ^4^K-herb Research Center, Korea Institute of Oriental Medicine, Daejeon, South Korea

**Keywords:** lobeglitazone, asthma, peroxisome proliferator-activated receptor, airway inflammation, mucus hypersecretion

## Abstract

Lobeglitazone (LB) is a novel agonist of peroxisome proliferator-activated receptor (PPAR)-α and γ that was developed as a drug to treat diabetes mellitus. We explored the ameliorative effects of LB on allergic asthma using a murine model of ovalbumin (OVA)-induced asthma. To boost the immune response of animals, OVA sensitization was performed on days 0 and 14. LB (250 or 500 μg/kg) was administered by oral gavage on days 18 to 23, and the OVA challenge was performed using an ultrasonic nebulizer on days 21 to 23. Plethysmography showed airway hyperresponsiveness (AHR) on day 24. LB treatment effectively decreased inflammatory cell recruitment, T-helper type 2 cytokines in the bronchoalveolar lavage fluid, and immunoglobulin (Ig) E in the serum of the animals with OVA-induced asthma, which was accompanied by a marked reduction in AHR. It also decreased airway inflammation, mucus hypersecretion, phosphorylation of nuclear transcription factor-kappa-B (NF-κB), and expression of activating protein (AP)-1 and mucin 5AC (MUC5AC). Overall, LB effectively attenuated the pathophysiological changes of asthma and its effects appear related to a reduction in the phosphorylation of NF-κB and the expression of AP-1. Thus, our results suggest that LB has a potential to treat allergic asthma.

## Introduction

Asthma is a widespread chronic airway disorder and its prevalence has continuously increased in modern society (Akinbami et al., 2015; Khorasanizadeh et al., 2017). It is also a chronic inflammatory diseases featured as variable airflow obstruction due to inflammatory responses, mucus production and airway hyperreactivity (Park et al., 2016). The pathogenesis of asthma is very complicated because of the various factors involved, such as cytokines, chemokines, growth factors, reactive oxygen species, T-cells and inflammatory cells (Park et al., 2016). Of these factors, increased T helper (Th)2 cytokines are believed to be a crucial pathophysiological cause of asthma, because they are closely associated with eosinophil recruitment, maturation and activation (Lee et al., 2010). In addition, the transcription factors activator protein (AP)-1 and nuclear factor-kappa B (NF-κB) are involved in the progression of inflammatory responses (McLeod et al., 2017). They are activated by various harmful stimuli, after which they translocate into the nucleus and bind to their promoter lesions. Eventually, the transcription factors produce proinflammatory mediators such as cytokines and chemokines (Zhou et al., 2014). Many experimental studies have described NF-κB and AP-1 as important therapeutic targets in asthma (Zhou et al., 2014; Schuliga, 2015).

Peroxisome proliferator-activated receptors (PPARs) are the nuclear receptor superfamily and have three subtypes, α, δ, and γ. All three subtypes are ligand-activated transcription factors (Karak et al., 2013). Although PPAR-α and -γ are known to regulate the expression of the genes involved in lipid metabolism, a previous study reported inhibition of airway inflammation by PPAR-α and -γ in a murine asthma model through inhibition of eosinophilia and lymphocyte influx into airways (Liu et al., 2015). Lobeglitazone (LB) is a novel dual agonist of PPAR-α and γ; it has a higher affinity for PPAR-γ than for PPAR-α, for which it has partial affinity, and is used for the management of type 2 diabetes mellitus (Kim et al., 2011; Lim et al., 2015). A recent study reported that LB reduced neointimal formation after balloon injury in rat carotid arteries by attenuating NF-κB phosphorylation (Lim et al., 2015). However, there are no studies on the protective effects of LB against allergic asthma.

Thus, we explored the ameliorative effects of LB using ovalbumin (OVA) induced asthma model. We also investigated the mechanism underlying the ameliorative effects of LB on asthma with a focus on its NF-κB-modulatory effect.

## Materials and Methods

### Animals

Female BALB/c mice (Specific-pathogen-free, 7 weeks old, 20–25 g, Koatech Co., Pyeongtaek, South Korea) were used after 1 week of quarantine and acclimatization. The mice were housed in polycarbonate cages under a controlled environment (temperature 22 ± 2°C and humidity 55 ± 5%). All procedures were granted by the Institutional Animal Care and Use Committee of Chonnam University (CNU IACUC-YBR-2016-19, Gwangju, Korea).

### Experimental Procedures

Ovalbumin induced asthma model was performed as described previously (Lee et al., 2010). Seven mice per mice were used in the experiment. The mice were treated with 20 μg OVA (Sigma-Aldrich, St. Louis, MO, United States) mixed with 2 mg aluminum hydroxide (Sigma-Aldrich) by intraperitoneal injection on days 0 and 14. One week after the final sensitization, OVA (1%, w/v, in PBS) challenge was performed for 1 h on days 21, 22, and 23. Dexamethasone (3 mg/kg, Dex, Sigma-Aldrich) and LO (250 μg/kg and 500 μg/kg, LB-0.25 and -0.5, respectively, Chong Kun Dang Pharm., Seoul, South Korea) were administered once daily by oral gavage from days 18 to 23. On day 24, airway hyperresponsiveness (AHR) in conscious and unrestrained mice was determined using whole-body plethysmography (OCP3000 instrument; Allmedicus, Seoul, South Korea). Bronchoalveolar lavage fluid (BALF) was obtained on day 25. Briefly, the mice were anesthetized via an intraperitoneal injection of Zoletil 50 (Virbac, France) and a tracheotomy was performed. The trachea was cannulated and the left bronchi were tied for histological experiments. Following instillation of ice cold PBS (0.5 mL) into the lungs, BALF was obtained using three times (total volume 1.5 mL). After the exclusion of dead cells through Trypan blue staining, the total inflammatory cell numbers were determined by counting the cells in at leat five squares of a hemocytometer. The differential cell count of the BALF was performed using Diff-Quik^®^ reagent (IMEB Inc., Deerfield, IL, United States).

### Assessment of Th2 Cytokines, Chemokine, and Immunoglobulin E Levels in BALF or Serum

T helper cytokines including interleukin (IL)-5 (R&D System, Minneapolis, MN, United States), IL-13 (R&D System), and mucin 5AC (MUC5AC; MyBioSource, San Diego, CA, United States) of BALF were measured by enzyme-linked immunosorbent assay (ELISA) kits. The total immunoglobulin E (IgE; BioLegend Inc., San Diego, CA, United States) level in the serum was determined by ELISA. The production of OVA-specific IgE in serum was evaluated using an ELISA kit (BioLegend Inc., San Diego, CA, United States). Specifically, 96-well microtiter plates were coated overnight with OVA (10 μg/mL in PBS-Tween-20). After incubation, the samples were added to each well and the plates were washed, blocked and incubated for an additional 2 h. The plates were then washed, horse-radish peroxidase (HRP)-conjugated goat anti-mouse IgE antibodies were added, and the plates were washed again. *o*-Phenylenediamine dihydrochloride (200 μL, Sigma-Aldrich) was then added, and the plates were incubated for 10 min in the dark. Absorbance was measured at 450 nm using an ELISA plate reader (Bio-Rad Laboratories, Hercules, CA, United States).

### Histology

For the histological examination, prior to lung removal, the left lung (which had not been lavaged) was filled intratracheally with 0.8% formalin and 4% acetic acid) and fixed in neutral buffered formalin [10% (v/v)]. The tissues were embedded, sectioned (4 μm), and stained with hematoxylin and eosin solution (Sigma-Aldrich) or the periodic acid-Schiff solution (IMEB Inc.). To investigate protein expression in lung tissue, we performed an immunohistochemical analysis. Paraffin-embedded sections were deparaffinized, dehydrated, washed with PBS containing 0.3% Triton X-100, and incubated for 10 min at room temperature with 10% goat serum to block non-specific staining. The slides were incubated overnight with primary mouse MUC5AC antibody that was used at a concentration of 1:100 dilution (Abcam). After incubating with the primary antibodies, the slides were washed and incubated with biotinylated secondary antibodies at 37°C for 1 h and then incubated with an avidin-biotin-peroxidase complex (Vector Laboratories, Burlingame, CA, United States) for 1 h at room temperature. The excess complex was removed and slides were washed with PBS prior to incubating in 0.05% diaminobenzidine (1:200, Millipore Co., Bedford, MA, United States) for 10 min. The slides were counterstained, rinsed with PBS to terminate the reaction, and protected with coverslips prior to microscopic examination. Quantitative analysis of histology was conducted using the IMT i-Solution software (IMT i-Solution Inc., Vancouver, BC, Canada).

### Immunoblotting

Lung tissues were homogenized with a tissue lysis/extraction reagent (Sigma-Aldrich, Carlsbad, CA, United States). The concentration of proteins in each sample was determined using Bradford reagent (Bio-Rad Laboratories, Hercules, CA, United States). Equal amounts of cellular proteins (30 μg) were resolved by 10% sodium dodecyl sulfate polyacrylamide gel electrophoresis (SDS–PAGE) and transferred onto a polyvinylidene fluoride (PVDF) membrane. The membrane was incubated in blocking solution (5% skim milk, Millipore Co., Bedford, MA, United States), followed by overnight incubation at 4°C with the appropriate primary antibodies, as follows: anti-p65 (Cell Signaling, Denver, MA, United States), anti-p-p65 (Cell Signaling) anti-MUC5AC (Abcam), anti-AP-1 (Cell Signaling) and anti-β-actin (Cell Signaling) antibodies. The blots were washed with Tris-buffered saline containing Tween 20 (TBST), and then incubated with a horseradish peroxidase (HRP)-conjugated secondary antibody (Jackson Immuno Research, West Grove, PA, United States) for 30 min at room temperature. The blots were washed again with TBST, and then, developed using an enhanced chemiluminescence kit (Thermo Scientific, San Diego, CA, United States). We evaluated the band expression values by ChemiDoc^TM^ (Bio-Rad, Hercules, CA, United States).

### Statistical Analysis

Results are expressed as means ± standard deviation values. Statistical significance was determined using analysis of variance followed by Dunnett’s adjustment. A *P-*value < 0.05 was considered as significant.

## Results

### Effects of LB on AHR

With an increase in methacholine concentration, the AHR of experimental animals increased compared to that in the normal controls (**Figure 1**). However, Dex-treated animals showed significantly declined AHR compared to that shown by the OVA group. In addition, the LB-treated animals exhibited a decline of AHR compared to that in the OVA group. These observations were noted in the high-dose LB group.

**FIGURE 1:** Effects of lobeglitazone (LB) on airway hyperresponsiveness (AHR) of OVA-challenged animals. AHR was measured using plethysmography 24 h after the final OVA challenge, in mice given various doses of methacholine (5–20 mg/ml). NC, normal control mice; OVA, OVA-sensitized/challenged mice; Dex, dexamethasone (3 mg/kg) + OVA-sensitized/challenged mice; LB-0.25 and –0.5, LB (250 μg/kg or 500 μg/kg, respectively) +OVA-sensitized/challenged mice. Values are expressed as mean ±*SD* (*n* = 6/group). ^#^Significantly different from NC, *P* < 0.05. ^∗^Significantly different from OVA, *P* < 0.05.

### Effects of LB on Inflammatory Cells Accumulation in the BALF From OVA Sensitized and Challenged Mice

The OVA sensitized and challenged animals exhibited the elevation of inflammatory cell counts including eosinophils, macrophages, lymphocytes and total cell counts compared to those in the normal controls (**Figure 2**). However, the Dex-treated animals showed the reduced counts of eosinophils, macrophage, lymphocytes, and total cells. These reductions were observed in the LB-treated animals. The low-dose LB animals (LB-0.25) exhibited a decline in eosinophil and total cell counts in comparison to those in the OVA sensitized and challenged mice. The high-dose LB animals (LB-0.5) exhibited a reduction in eosinophil, macrophage and total cell counts.

**FIGURE 2:** Effects of lobeglitazone (LB) on the number of inflammatory cells in BALF from OVA challenged animals. Cells were isolated via centrifugation and stained with Diff-Quick stain reagent. NC, normal control mice; OVA, OVA-sensitized/challenged mice; Dex, dexamethasone (3 mg/kg) + OVA-sensitized/challenged mice; LB-0.25 and –0.5, LB (250 μg/kg or 500 μg/kg, respectively) + OVA-sensitized/challenged mice. Values are expressed as mean ±*SD* (*n* = 6/group). ^#^Significantly different from NC, *P* < 0.05. ^∗^Significantly different from OVA, *P* < 0.05.

### Effects of LB on Th2 Cytokines and MUC5AC Levels in the BALF and Ig E in the Serum From OVA Sensitized and Challenged Mice

The levels of IL-5 (55.4 ± 11.5 pg/mL) and IL-13 (62.4 ± 11.7 pg/mL) were elevated in the OVA sensitized and challenged animals compared to those in the normal controls (**Figures 3A,B**, respectively). However, the LB-treated animals exhibited a decline in IL-5 (33.9 ± 6.6 pg/mL in 0.25 mg/kg group and 31.2 ± 7.6 pg/mL in 0.5 mg/kg group) and IL-13 (48.1 ± 9.1 pg/mL in 0.25 mg/kg and 43.2 ± 9.3 pg/mL in 0.5 mg/kg group) levels in comparison to those in the OVA sensitized and challenged animals. Similarly, the OVA sensitized and challenged animals showed the elevated MUC5AC production (0.39 ± 0.04 absorbance) compared to that in the normal controls. On the other hand, the LB-treated animals showed a decrease in MUC5AC production (0.33 ± 0.04 absorbance in 0.25 mg/kg group and 0.28 ± 0.04 absorbance in 0.5 mg/kg group) compared to that in the OVA sensitized and challenged animals (**Figure 3C**). Consistent with the results of the BALF analysis, the OVA sensitized and challenged animals showed the increased total Ig E (822.6 ± 172.2 ng/mL) and OVA-specific Ig E (97.83 ± 24.8 ng/mL) levels in comparison to those in the normal controls, whereas the LB-treated animals showed a decreases (IgE : 609.8 ± 87.7 ng/mL in 0.25 mg/kg group and 515.0 ± 144.8 ng/mL in 0.25 mg/kg group, OVA-specific IgE : 75.0 ± 18.7 ng/mL in 0.25 mg/kg group and 60.9 ± 14.2 ng/mL in 0.5 mg/kg group) in comparison to those in the OVA sensitized and challenged animals (**Figures 3D,E**, respectively).

**FIGURE 3:** Effects of lobeglitazone (LB) on IL-5, IL-13, and MUC5AC levels in BALF and total IgE and OVA-specific IgE levels in serum from OVA-challenged animals. IL-5, MUC5AC, total IgE, and OVA-specific IgE levels were determined using ELISA Kit. **(A)** IL-5 in BALF, **(B)** IL-13 in BALF, **(C)** MUC5AC in BALF, **(D)** Total IgE in serum, **(E)** OVA-specific IgE. NC, normal control mice; OVA, OVA-sensitized/challenged mice; Dex, dexamethasone (3 mg/kg) + OVA-sensitized/challenged mice; LB-0.25 and –0.5, LB (250 μg/kg or 500 μg/kg, respectively) + OVA-sensitized/challenged mice. Values are expressed as mean ± *SD* (*n* = 6/group). ^#^Significantly different from NC, *P* < 0.05. ^∗^Significantly different from OVA, *P* < 0.05.

### Effects of LB on Airway Inflammation and Mucus Production in Lung Tissue of OVA Sensitized and Challenged Mice

As shown in **Figures 4A,B**, the OVA sensitized and challenged animals showed inflammatory cell accumulation into lung tissue compared to that in the normal controls. However, the LB-treated animals exhibited the attenuation of inflammatory cell accumulation into lung tissue. Furthermore, the OVA sensitized and challenged animals showed a mucus overproduction in the bronchial lesion whereas the LB-treated animals exhibited a significant decline of mucus production (**Figures 4A,C**). Consistent with the results obtained for mucus production, MUC5AC expression also decreased in the LB-treated animals compared to that in the OVA sensitized and challenged animals (**Figures 4A,D**).

**FIGURE 4:** Effects of lobeglitazone (LB) on airway inflammation, mucus production, and MUC5AC expression in lung tissue from OVA-challenged animals. **(A)** Representative figure of airway inflammation, mucus production, and MUC5AC expression in lung tissue. Quantitative analysis of airway inflammation **(B)**, mucus production **(C)**, and MUC5AC expression **(D)** in lung tissue, respectively. NC, normal control mice; OVA, OVA-sensitized/challenged mice; Dex, dexamethasone (3 mg/kg) + OVA-sensitized/challenged mice; LB-0.25 and –0.5, LB (250 μg/kg or 500 μg/kg, respectively) + OVA-sensitized/challenged mice. Values are expressed as mean ±*SD* (*n* = 6/group). ^#^Significantly different from NC, *P* < 0.05. ^∗^Significantly different from OVA, *P* < 0.05.

### Effects of LB on p65 Phosphorylation and Expression of AP-1 and MUC5AC

The OVA sensitized and challenged animals showed significantly increased p65 phosphorylation in lung tissue compared to that shown by the normal controls (**Figures 5A,B**). However, the LB-treated animals exhibited a significant decline of p65 phosphorylation. Similarly, the expression of AP-1 and MUC5AC increased in the OVA sensitized and challenged animals compared to that in the normal controls. In contrast, the LB-treated animals showed a decline in the expression of AP-1 and MUC5AC.

**FIGURE 5:** Effects of lobeglitazone (LB) on the expression of NF-κB, AP-1 and MUC5AC expression of lung tissue from OVA-challenged animals. **(A)** Gel images showing protein expression. **(B)** Relative expression ratio of protein. NC, normal control mice; OVA, OVA-sensitized/challenged mice; Dex, dexamethasone (3 mg/kg) + OVA-sensitized/challenged mice; LB-0.25 and –0.5, LB (250 μg/kg or 500 μg/kg, respectively) + OVA-sensitized/challenged mice. Values are expressed as mean ± *SD* (*n* = 6/group). ^#^Significantly different from NC, *P* < 0.05. ^∗^Significantly different from OVA, *P* < 0.05.

## Discussion

We explored the therapeutic effects of LB, a novel dual agonist of PPAR-α and γ, on airway inflammation and mucus hypersecretion in OVA sensitized and challenged mice and its possible mechanism of action. LB effectively decreased AHR, inflammatory cell infiltration, levels of Th2 cytokines and MUC5AC of BALF with the decline of total Ig E and OVA-specific Ig E levels in the serum of OVA sensitized and challenged animals. Furthermore, LB treatment decreased airway inflammation and mucus production in OVA sensitized and challenged animals. It also reduced p65 phosphorylation and the expression of AP1 and MUC5AC in the lung tissue of OVA sensitized and challenged animals.

T helper cytokines are regarded as a critical factor in the development of allergic asthma represented by AHR, eosinophilic inflammation, and mucus hypersecretion. These cytokines promote inflammatory cell infiltration, Ig E production, and mucus overproduction and are involved in the production of other proinflammatory mediators such as chemokines, inflammatory proteins, and proteolytic enzymes (Schatz and Rosenwasser, 2014). In particular, eosinophil infiltration into the airways results from the production of IL-5 and IL-13, which play important roles in the proliferation, activation, and migration of eosinophils (Lee et al., 2010). In this work, LB significantly decreased the levels of Th2 cytokines in OVA sensitized and challenged animals, which was accompanied by a decline of eosinophils count, total IgE and OVA-specific IgE. These results were strongly supported by the findings of the histological analysis. LB treatment effectively decreased inflammatory responses and mucus production in OVA sensitized and challenged animals. These results suggest that LB exhibits protective effects against asthmatic responses by reducing Th2 cytokine levels.

Proinflammatory cytokines developed inflammatory responses through the activation of various inflammatory signaling pathways (Lee et al., 2010). In particular, NF-κB expression significantly increased in asthmatic animals (Schuliga, 2015). Phosphorylation of NF-κB induced by various factors is considered as a limiting step in the progression of inflammatory responses and mucus production (Park et al., 2017). In the progression of inflammatory responses, NF-κB acts as a transcription factor. p65 is a subunit of NF-κB with p50 and is phosphorylated by various stimuli. Phosphorylated p65 translocated into the nucleus and then it binds to the promotor region and produces various inflammatory mediators resulting in asthmatic responses (Cai et al., 2018). AP-1 also is considered as a major activator of inflammatory genes. According to previous studies, AP-1 expression was elevated in RAW264.7 cells by lipopolysaccharide treatment and induced the production of proinflammatory cytokines (Han et al., 2017; Ahn et al., 2018). Because of this evidence, NF-κB and AP-1 are considered potential therapeutic targets in various inflammatory diseases (Lee et al., 2017; McLeod et al., 2017). Furthermore, the expression of NF-κB and AP-1 leads to the production of MUC5AC that are major gel-forming mucins in airway secretions (Lee et al., 2017; Ding et al., 2018). Particularly, MUC5AC is well-kwon as a main component of airway mucus and associated with airflow limitation and AHR in patients with asthma (Evans et al., 2015). Thus, modulation of the NF-κB and AP-1 pathways would be a potential therapeutic target to treat asthma. In this work, the OVA sensitized and challenged animals showed the increased NF-κB phosphorylation and AP-1 expression with the elevation of MUC5AC expression in the lung tissue. However, LB treatment showed the reductions in NF-κB phosphorylation and AP-1 expression accompanied by a decline in MUC5AC expression. These findings indicated that LB attenuated the airway inflammation and mucus production in OVA sensitized and challenged animals through the downregulation of NF-κB phosphorylation and AP-1 expression.

## Conclusion

In conclusion, LB attenuated asthmatic signs including airway inflammation and mucus hypersecretion in OVA sensitized and challenged animals. These effects were closely related to the downregulation of NF-κB phosphorylation and AP-1 expression in lung tissue. Thus, LB may effectively inhibit OVA-induced asthma.

## Author Contributions

N-RS, I-SS, and J-SK conceived and designed the experiments. N-RS, S-HP, and J-WK performed the experiments. I-SS and J-SK analyzed the data. Y-KC, I-CL, and J-CK contributed to the reagents, materials, and analysis tool. N-RS wrote the paper.

## Conflict of Interest Statement

The authors declare that the research was conducted in the absence of any commercial or financial relationships that could be construed as a potential conflict of interest.
